This article has been retracted.

# The effect of secukinumab treatment for psoriasis on serum cytokines and correlation with disease severity

**DOI:** 10.1111/srt.13405

**Published:** 2023-07-06

**Authors:** Lan‐Tu‐Ya Wu, Zhu‐Hui Qiao, Jia‐Bin Tian, Jia‐Lin Lin, Su‐Chun Hou, Xiao‐Ming Liu

**Affiliations:** ^1^ School of Pharmaceutical Science, Health Science Center Shenzhen University Shenzhen China; ^2^ Department of Dermatology The University of Hong Kong‐Shenzhen Hospital Shenzhen China; ^3^ Health Science Center Shenzhen University Shenzhen China

**Keywords:** DEFB2, GRO α (CXCL1), IFN‐ γ, IL‐1 β, IL‐10, IL‐12, IL‐13, IL‐17A, IL‐18, IL‐1RA, IL‐22, IL‐23, IL‐6, PCT, Psoriasis, secukinumab, TARC, TNF‐ α, VEGF‐A

## Abstract

**Objective:**

To investigate the effects of secukinumab treatment for psoriasis on different functional cytokines and inflammatory mediators in patients’ serum

**Methods:**

Enzyme‐linked immunosorbent assay was used to detect interleukin (IL)‐1β and IL‐1RA associated with intrinsic immunity; IL‐6, IL‐18, and growth regulated oncogene alpha (GROα) associated with neutrophils; IL‐12, tumour necrosis factor (TNF)‐α, and interferon (IFN)‐γ associated with Th1; IL‐23, IL‐17A, and IL‐22 associated with Th17; Thymus activation regulated chemokine (TARC), IL‐13, and defensin beta 2 (DEFB2) associated with Th2; Vascular endothelial growth factor (VEGF)‐A and IL‐10 associated with angiogenesis; and IFN‐γ associated with sepsis in the peripheral blood of 12 patients with common psoriasis treated with secukinumab and 15 healthy controls. IL‐23, IL‐17A, IL‐22 associated with Th17; TARC, IL‐13, DEFB2 associated with Th2; VEGF‐A, IL‐10 associated with angiogenesis and procalcitonin (PCT) associated with sepsis. The differences in expression of the above cytokines before and after treatment and the correlation with psoriasis disease severity［Psoriasis Area Severity Index(PASI) score］, age, and disease duration were analyzed.

**Results:**

The mean PASI score of the enrolled patients with moderate to severe psoriasis was 21.6 ± 11.0 before treatment and decreased to below 1 after treatment. Serum IL‐6; IL‐18, GROα, IFN‐γ, TNF‐α, VEGF‐A, and IL‐17A were significantly higher than normal. And IL‐17A and IFN‐γ were positively correlated with disease duration and age, and IL‐18 was positively correlated with PASI score. The expression levels of IL‐6, GROα, VEGF‐A, IFN‐γ, TNF‐α, IL‐17A and IL‐23 were significantly lower after secukinumab treatment compared with those before treatment, but the expression levels of IFN‐γ, VEGF‐A, TARC, IL‐13, and DEFB2 were still significantly higher than those of normal subjects after treatment

**Conclusions:**

secukinumab clears skin lesions by antagonizing IL‐17A and simultaneously decreasing the expression levels of IL‐6, GRO α, VEGF‐A, IFN‐γ, TNF‐α, IL‐17A, and IL‐23.

## 1 INTRODUCTION

Psoriasis is a chronic, relapsing inflammatory disease. It mainly affects the skin and joints and can be combined with co‐morbidities such as metabolic syndrome and cardiovascular diseases. The manifestations of skin plaques, joint inflammation and co‐morbidities are associated with the infiltration of immune cells and secreted cytokines in the blood and tissues. Currently, the pathogenesis of psoriasis is focused on the IL‐23‐Th17 axis, and the related cytokines IL‐23, IL‐17A, and IL‐22 play a key role in the pathogenesis of psoriasis, and secukinumab, which antagonizes IL‐17A, has shown very good efficacy in the clinical treatment of psoriasis. However, there are also multiple cytokines involved in the immune circuit of psoriasis pathogenesis. For example, IL‐1β, IL‐1RA, IL‐6, IL‐18, GROα associated with intrinsic immunity and neutrophils; VEGF‐A, IL‐10 associated with angiogenesis; IFN‐γ, TNF‐α, IL‐12 associated with Th1; PCT associated with sepsis, etc. Some studies have shown that these cytokines are also involved in the pathogenesis of psoriasis.^1^ However, the relationship with disease severity and changes before and after drug treatment are not fully established. Psoriasis can present with eczema‐like changes, and it is uncertain whether Th2‐associated TARC, DEFB2, and IL‐13 are also involved in the pathogenesis of psoriasis. In this study, we analyzed the changes of 17 cytokines in serum before and after treatment in 12 patients with moderate‐to‐severe psoriasis treated with secukinumab to assess the relationship between these cytokines and psoriasis severity andtreatment, and to investigate the possible mechanisms for the treatment of psoriasis with secukinumab.

## 2 RESULTS

### 2.1 Differences in the expression of different cytokines in serum of patients with moderate to severe psoriasis

Serum expression of IL‐6, IL‐18, GROα associated with intrinsic immunity and neutrophils; IFN‐γ, TNF‐α associated with Th1; VEGF‐A associated with angiogenesis; IL‐17A associated with Th17; TARC, DEFB2, IL‐13 associated with Th2 were significantly higher than normal in patients with moderate to severe psoriasis (*p* < 0.05). The expression levels of IL‐12, IL‐23, PCT, and IL‐1β were greater than those of normal subjects before treatment, but not statistically significant. The expression levels of serum IL‐22, IL‐1RA, and IL‐10 in patients with moderate to severe psoriasis were lower than normal, and the decreased level of IL‐22 was significantly different compared with normal subjects (*p* < 0.01) (Table 1, Figures 1, 2, 3, 4, 5, 6).

**TABLE 1:** General information of patients with psoriasis.

Number	Gender	Age	BMI	Course of disease (year)	PASI score before treatment	BSA score before treatment	PASI score after treatment	BSA score after treatment
1	M	24	23	5	13.6	18	0.1	0.5
2	M	28	33	10	27.6	60	0	0
3	F	31	23	15	35.2	50	0	0
4	M	34	28	15	35	20	0	0
5	F	35	20	20	9.3	13	0	0
6	F	38	22	20	41.3	70	0	0
7	M	35	24	5	25	50	0	0
8	F	41	27	20	19.8	40	0	0
9	M	40	25	25	14	40	0	0
10	M	49	24	15	16.8	12	0.6	1
11	F	24	34	15	10.8	12	0.7	2
12	M	41	27	10	10.8	7	0.4	1

**FIGURE 1:** Expression levels of IL‐1ra, IL‐1β, L‐6 cytokines in serum of psoriasis patients before and after treatment and in normal subjects.

**FIGURE 2:** Expression levels of IL‐18, GRO‐α, PCT in serum of psoriasis patients before and after treatment and in normal subjects.

**FIGURE 3:** Expression levels of VEGF‐A, IL‐10 cytokines in serum of psoriasis patients before, after treatment and in normal subjects.

**FIGURE 4:** Levels of IFN‐γ, TNF‐α, IL‐12 cytokine expression in serum of psoriasis patients before and after treatment and in normal subjects.

**FIGURE 5:** Levels of IL‐17A, IL‐22, IL‐23 cytokine expression in serum of psoriasis patients before and after treatment and in normal subjects.

**FIGURE 6:** Expression levels of DEFB2, IL‐13, TARC in serum of psoriasis patients before and after treatment and in normal subjects.

### 2.2 Chages in serum cytokines after secukinumab treatment in patients with moderate‐to‐severe psoriasis

Serum levels of neutrophil‐related IL‐6 and IL‐1β; GROα and IL‐18; angiogenesis‐related VEGF‐A and IL‐10; Th1‐related IFN‐γ, TNF‐α and IL‐12; Th17‐related IL‐17A and IL‐23; Th2‐related TARC, DEFB2 and IL‐13; and sepsis‐related PCT were reduced in patients with moderate‐to‐severe plaque psoriasis treated with secukinumab. Th2‐related TARC, DEFB2, IL‐13; and sepsis‐related PCT levels were all reduced compared with those before treatment. The levels of IL‐6, GROα, VEGF‐A, IFN‐γ, TNF‐α, IL‐17A and IL‐23 were significantly lower after treatment than before treatment, with significant differences (*p* < 0.05, *p* < 0.01). Only IL‐1RA and IL‐22 serum levels were slightly higher after treatment than before treatment, but there was no statistically significant difference (*p* > 0.05) (Table 1, Figures 1, 2, 3, 4, 5, 6).

### 2.3 Comparison of serum cytokine levels in psoriasis patients with normal subjects after secukinumab treatment

Serum angiogenesis‐related VEGF‐A; Th1‐related IFN‐γ and Th2‐related DEFB2 serum expression levels remained significantly higher in patients with moderate‐to‐severe psoriasis after secukinumab treatment than in normal subjects. the expression levels of VEGF‐A and IFN‐γ were significantly lower after secukinumab treatment than before treatment (Table 1, Figures 1, 2, 3, 4, 5, 6).

### 2.4 Correlation of different cytokine expression levels with disease duration and disease severity

Both IL‐17A and TNF‐α were positively correlated with disease duration and age; IL‐18 was positively correlated with PASI; and TARC was correlated with gender, with males significantly higher than females. Other cytokines did not correlate with disease severity (Table 1, Figure 7).

FIGURE 7Correlation of different cytokine expression levels with disease duration and disease severity.

(1) IL‐17A was positively correlated with disease duration, *p* = 0.012; (2) IL‐17A was positively correlated with age, *p* = 0.035; (3) TNF‐α was positively correlated with disease duration, *p* = 0.01; (4) TNF‐α was positively correlated with age, *p* = 0.02; (5) TARC was correlated with gender, significantly higher in men than in women, *p* = 0.008; (6) IL‐ 18 was positively correlated with PASI score, *p* = 0.033

## 3 DISCUSSION

Psoriasis is a common chronic inflammatory disease characterized by excessive proliferation of keratinocytes and abnormal infiltration of effector T cells, dendritic cells, neutrophils, and macrophages. The pathogenesis of psoriasis involves a complex immune network formed by the interaction between multiple cell types and the cytokines secreted by them.^1^ The interaction between innate and adaptive immunity, epithelial and vascular systems maintains the inflammatory environment of psoriasis. The results of this study showed that serum IL‐6 associated with neutrophils; IL‐18, CXCL1; IFN‐γ, TNF‐α associated with Th1; VEGF‐A associated with angiogenesis; and IL‐ associated with Th17 proliferation in patients with moderate to severe psoriasis (PASI score mean 21.6 ± 11.0,BSA score mean 32.67 ± 21.58) 17A were all significantly higher than those in normal subjects. Moreover, IL‐17A and IFN‐γ were positively correlated with the disease duration and patient's age, and IL‐18 was positively correlated with the disease severity PASI score. This further confirms the involvement of multiple immune cells and associated cytokines in the pathogenesis of psoriasis.

It is now generally accepted that the IL‐23‐Th17 axis plays a key role in the pathogenesis of psoriasis. Elevated levels of IL‐17 in lesions, serum and nonlesioned skin of patients with psoriasis are positively correlated with disease severity.^2^, ^3^, ^4^, ^5^ Secukinumab, a fully human IgG1 monoclonal antibody that selectively antagonizes IL‐17A, has shown very good efficacy in the clinical treatment of psoriasis. However, the mechanism by which the drug eliminates skin lesions is not fully understood. Available studies suggest that the onset of psoriasis is preceded by the activation of innate immunity, in which the skin receives external stimuli that cause a complex of LL37 and its own DNA to activate dermal plasmacytoid dendritic cells (pDCs) via the Toll‐like receptor signaling pathway. pDCs release the inflammatory mediators interferon α and β, which stimulate myeloid DCs to secrete additional proinflammatory mediators IL‐12, IL‐23, and TNF‐α. These natural immune mediators stimulate the  overproliferation of key T lymphocyte subsets such as Th1, Th17 and Th22, releasing additional cytokines and chemokines such as IL‐17, IL‐22, TNF‐α, and IFN‐γ, triggering a cascade response in psoriasis.^1^, ^6^ Stressed keratin‐forming cells also secrete IL‐1 and IL‐6.^7^ IL‐17A also stimulates the expression of antimicrobial peptides (AMPs), including β‐defensins and members of the S100A family, activates the production of multiple chemokinessuch as CXCL6, CCL20, CXCL1, CXCL2, CXCL3, CXCL5, and CXCL8/IL‐8, and stimulates neutrophil recruitment and activation.^1^ This suggests that IL‐6, CXCL1, TNF‐α, IL‐17A, and IL‐23 all play important roles in the pathogenesis of psoriasis. It has been suggested that IL‐17A blockers clear lesions by altering psoriasis gene expression.^13^ Merlijn et al.^8^ examined several markers of angiogenesis and tissue remodeling in serum samples from 20 patients with active peripheral spondyloarthritis (SpA before and after secukinumab treatment. Serum IL‐6, IL‐31, VEGF‐A, IL‐33, TNF‐α were also found to be significantly reduced after anti‐IL‐17A treatment. The mean PASI score of the patients selected for this study was 21.6 ± 11.0 before treatment, and the lesions were nearly completely resolved after treatment (PASI < 1). The expression levels of serum cytokines IL‐6, CXCL1, VEGF‐A, IFN‐γ, TNF‐α, IL‐17A, and IL‐23 were significantly lower after treatment compared with those before treatment. Review of the literature revealed that all of these cytokines were associated with IL‐17. Located upstream and downstream of IL‐17A, the expression of these cytokines and inflammatory mediators was simultaneously suppressed when IL‐17A was inhibited. It can be assumed that IL‐17A antagonists achieve clearance of skin lesions by inhibiting the inflammatory cascade response to IL‐17A.^9^

The results of this study showed that IFN‐γ and VEGF‐A expression levels were significantly higher than normal in psoriasis patients before treatment and decreased significantly after secukinumab treatment, but the levels remained significantly higher than normal after treatment. IFN‐γ is the only member of the type II interferon family. In psoriasis Th1 cells are a potential source of IFN‐γ. Previously, the Th1 pathway was considered to be the main pathogenic pathway in psoriasis.^1^ However, with the introduction of IL‐17A antagonists, the potential role of IFN‐γ seems to have become less important. According to clinical, histological and molecular markers, selective blockade of IL‐23‐induced IL‐17A leads to complete recovery from psoriasis; nevertheless, IFN‐γ has a role in promoting the release of IL‐23, IL‐1 and chemokines CXCL10 and CXCL11, as well as the expression of dendritic cells, T cells, keratinocytes and endothelial cell adhesion molecules, which can promote inflammatory cells to lesion recruitment of plaques. However, direct blockade of IFN‐γ with neutralizing antibodies was not therapeutically effective in patients with psoriasis, suggesting that IFN‐γ is not directly involved in the development of psoriasis.^1^ The results of the present study IL‐17A antagonists, although significantly reducing IFN‐γ levels, remained higher than normal after treatment, indicating that there is no direct relationship between elevated IFN‐γ levels and skin lesions.

VEGF‐A mediates angiogenesis and is upregulated in plaque and plasma expression in psoriasis patients. Transgenic expression of VEGF‐A in experimental models leads to skin lesions characteristic of psoriasis.^10^VEGF‐A and its receptors VEGFR‐1 and VEGFR‐2 mediate inflammatory angiogenesis in psoriasis, leading to vasodilation and enlargement, endothelial proliferation and hyperpermeability.^11^ The present study also showed that VEGF‐A is involved in the pathogenesis of psoriasis and that IL‐17A antagonists, although reducing VEGF‐A expression levels, do not normalize them, Luengas‐Martinez et al.^10^ suggested that a subset of psoriasis patients is prone to high levels of VEGF‐A and that they are most likely to benefit from anti‐VEGF‐A therapy, which provides an opportunity for personalized treatment.

Chen et al.^12^ applied fluorescent quantitative polymerase chain reaction (PCR) and gene clustering analysis to study peripheral blood and lesion tissues in 40 patients with psoriasis and 20 patients with atopic dermatitis (AD) and found two distinct clusters of psoriasis, both of which showed high Th17 activity. However, one group (six of the 40 psoriasis patients) had an increased Th2 component in the lesion tissues. This group of patients with psoriasis had significantly higher expression of IL‐4, IL‐13, IL‐25, IL‐31, and thymic stromal lymphopoietin (TSLP) genes compared to patients with AD. In this study, we found that the expression of Th2‐related TARC, DEFB2, and IL‐13 was significantly increased in the serum of patients with moderate‐to‐severe psoriasis and was not significantly decreased after secukinumab treatment, especially DEFB2, whose serum expression level remained significantly higher than normal after secukinumab treatment. It indicates that Th2 and related cytokines may be involved in the pathogenesis of psoriasis and do not respond significantly to treatment with IL‐7A antagonists.

## 4 MATERIALS AND METHODS

### 4.1 Types of cytokines tested

Sepsis‐related: PCT; intrinsic immune and neutrophil‐related: IL‐1β, IL‐1ra, IL‐6, IL‐18, GROα; Th1 cell‐related: IFN‐γ, IFN‐γ, IL‐12; angiogenesis‐related: VEGF‐A, IL‐10; Th17‐related: IL‐23, IL‐17A, IL‐22; Th2‐related: TARC, DEFB2, IL‐13.

### 4.2 Reagents and equipments

ELIASA kit is from Wuhan Elabscience; Enzyme microplate analyzer (Bethen, USA).

### 4.3 Patients and normal controls

Twelve patients with moderate‐to‐severe psoriasis were obtained from the dermatology outpatient clinic of the University of Hong Kong Shenzhen Hospital, including seven males and five females; age ranged from 24–49 years, with a median age of 35 years; disease duration ranged from 5–25 years, with a median disease duration of 15 years, before treatment was the time of the first dose, and after treatment was the time of complete or near‐complete regression of the lesions (PASI < 1): psoriasis lesion severity index PASI scores ranged from 9.3‐41.3, with a mean of 21.6 ± 11.0, and BSA scores ranged from 7–70, with a mean of 32.67 ± 21.58. Cases met the following criteria: (1) clinically and pathologically confirmed psoriasis; (2) patients who had not used biologics or traditional systemic therapy within 3 months; (3) no co‐morbidities such as diabetes, obesity, hyperlipidemia, cardiovascular disease, etc. (Table 1). (See Table 1 for details). Fifteen cases of healthy individuals matched for sex and age were also selected as controls, and the general information of the two groups was significantly different, as shown in Table 1.

### 4.4 Methods

The cytokines in the serum were detected by enzyme‐linked immunosorbent assay (ELISA), which was operated strictly according to the instructions of ELISA kit, and finally the OD value of each well was measured at 450‐nm wavelength of the enzyme calibrator, and the concentration of each cytokine in the serum was calculated according to the standard curve.

### 4.5 Statistical analysis

All data were analyzed using the Statistical Package for Social Sciences (SPSS) 26 program on the computer. All data are given as mean ± standard deviation. Wilcoxon signed rank test was used for pretreatment and posttreatment, Mann–Whitney *U* test for patients and healthy controls, and Spearman rank correlation test was used to assess correlations. *p‐*Value < 0.05 was considered statistically significant.

## 5 CONCLUSIONS

Secukinumab cleared skin lesions by antagonizing IL‐17A and reducing the expression levels of IL‐6, CXCL1, VEGF‐A, IFN‐γ, TNF‐α, IL‐17A, and IL‐23.

## CONFLICT OF INTEREST STATEMENT

The authors declare no conflict of interest.

### ETHICS STATEMENT

The study was conducted in accordance with the Declaration of Helsinki, and approved by the Ethics Committee of Medical Research Ethics Committee of The University of Hong Kong Shenzhen Hospital (protocol code: 伦［2019］181, date of approval:20190527). Written informed consent has been obtained from the patients to publish this paper.

## Data Availability

The data that support the findings of this study are available from the corresponding author upon reasonable request.
